The article "Application of Accelerated Rehabilitation Surgery in Gastrointestinal Surgery" was retracted in 2023. Reasons: signs of a paper mill; compromised peer review; unreliable results or conclusions.

# Application of Accelerated Rehabilitation Surgery in Gastrointestinal Surgery

**DOI:** 10.1155/2021/2968347

**Published:** 2021-12-28

**Authors:** Ke Liu, Yonghong Wang, Jun Wang, Na Luo, Juan Gong, Jian Wang, Bing Chen

**Affiliations:** People's Hospital of Leshan, Leshan, 614000 Sichuan, China

## Abstract

Adding timely rehabilitation surgery is an optimized perioperative measure that can reduce physical stress, reduce surgical risks, and postoperative complications and promote the recovery of organ function. Therefore, it is of great value to study its application in gastrointestinal surgery (GS). To this end, this article applies retrospective analysis and statistical methods to conduct targeted investigations and studies on GS patients. The results of the survey showed that 26.7% of patients were effective in ARS and 40% were effective in treatment. Compared with traditional treatment methods, its effective treatment rate is 13.4% higher.

## 1. Introduction

Improving the quality of medical services and improving the treatment effect of surgical patients are issues that surgeons have been paying attention to and thinking about. With the continuous advancement of modern surgical technology, there is more and more evidence from corroborative medicine showing that many traditional perioperative concepts are constantly being updated because they are not conducive to the recovery of patients. And ARS is a kind of perioperative period. Early surgery is limited to simple manual methods, such as abscess drainage, tumor resection, and trauma suture. Therefore, surgery is an operation that destroys tissue integrity (incision) or restores (sutures) the tissue whose integrity is damaged. With the development of surgery, the field of surgery is expanding and can be performed in any part of the human body. The applied instruments are also constantly updated, such as a scalpel, including an electric knife, microwave knife, ultrasonic knife, and laser knife.

There are many theoretical results in the application of ARS in GS. For example, Laizhi et al. explored the clinical effect of acute pancreatitis without gastrointestinal decompression based on the concept of ARS [1]. Weiwei and Yuli said that rapid rehabilitation surgery is a novel medical concept that can be applied to many types of surgery. The safety of perioperative use is high, which can improve the overall satisfaction of patients to a certain extent [2]. Qin believes that applying the concepts and measures of ARS to the care of patients with gastric cancer can accelerate the recovery of gastrointestinal function after surgery, shorten the hospital stay, and improve patient satisfaction [3]. Therefore, the research on gastrointestinal treatment in ARS is a research for the benefit of mankind, which can promote the acceleration of a patient's rehabilitation and functional recovery. The differential diagnosis of gastrointestinal diseases includes ultrasound scanning, which is suitable for the local section of organs. The panoramic observation is not as good as X-ray barium meal examination and endoscopy. The morphology and color of mucosa were not as good as X-ray barium examination and endoscopy. The detection rate of small ulcers, superficial lesions, and functional lesions is low, and the rate of missed and misdiagnosis is high.

The article "Application of Accelerated Rehabilitation Surgery in Gastrointestinal Surgery" was retracted in 2023. Reasons: signs of a paper mill; compromised peer review; unreliable results or conclusions.

This article first studies some basic knowledge of ARS. The second study is the perioperative management of GS. Then, the gastrointestinal surgical treatment was described in detail, and the economic benefits of ARS were analyzed. Finally, experiments were conducted on gastrointestinal patients, data were obtained, and conclusions were sorted and summarized. X-ray examination mainly depends on radiography, including gastrointestinal barium meal examination, colon barium enema examination, stomach gas barium double contrast examination, small intestine double contrast examination, and colon double contrast examination. Multiphasic gastrography and colonography should still be the ideal primary examination method for gastrointestinal diseases.

## 2. Application of Accelerated Rehabilitation Surgery in Gastrointestinal Surgery

### 2.1. Accelerated Rehabilitation Surgery

The concept of accelerated rehabilitation surgery (ERAS) is the extensive application of a series of optimized perioperative measures, supplemented by medical evidence, to reduce the psychological and physical burden of surgical trauma, reduce surgical complications, and quickly restore various organic functions. Shorten the time of surgery and hospitalization, improve the treatment effect, accelerate the recovery of patients, and ultimately achieve the goal of improving the quality of medical services [4, 5].

As a new surgical concept, it aims to reduce the body's response to surgery and trauma pressure through a series of evidence-based perioperative optimization measures to speed up recovery. It is the synergistic effect produced by a series of effective, optimized and comprehensive measures. The basic idea is to reduce trauma and stress, maintain a stable environment in the body, ensure normal physiological functions of the body, and promote patient recovery. The ERAS team is composed of multidisciplinary personnel, including surgeons, anesthesiologists, and nurses, who work closely with each other to ensure the implementation and implementation of accelerated rehabilitation measures [6, 7].

The article "Application of Accelerated Rehabilitation Surgery in Gastrointestinal Surgery" was retracted in 2023. Reasons: signs of a paper mill; compromised peer review; unreliable results or conclusions.

It has different processing methods in three stages. In preoperative education for patients, patients without clear gastrointestinal disorders are given a certain sugar load before surgery instead of conventional fasting water. Preoperative gastrointestinal decompression tube indwelling is no longer a routine. Minimally invasive techniques and the concept of damage control in surgery were applied. Attention is paid to heat preservation measures during surgery. General intravenous anesthesia with rapid onset and relatively simple operation is no longer selected for anesthesia, but epidural combined with general anesthesia. The more opioids are used for pain relief. More and more cautious, postoperative patient-controlled epidural analgesia combined with nonsteroidal analgesia is favored by anesthesiologists. Oral feeding or enteral nutrition after surgery is no longer waiting after intestinal ventilation. Require patients to take the initiative to rehabilitate and exercise in the early postoperative period. Remove various catheters such as abdominal drainage tubes and urinary catheters as soon as possible, apply antibiotics appropriately, and give antiemetics [8, 9]. Because of its own operation characteristics, traditional surgery will inevitably bring great trauma to patients while treating diseases. Not only the wound is large, the operation time is long, the hospital stay is long, the complications are large, and the recovery is slow, but also it is difficult to ensure the normal function of uterus and ovary, and the postoperative pain is often unbearable. The trauma itself can have serious consequences for patients. Minimally invasive technology is characterized by no operation, safety and ease, no pain during operation, short operation time, short hospital stay, minimal trauma to patients, no complications, and fast postoperative recovery, which is the biggest difference from traditional surgery.

With the development of surgical technology and the continuous improvement of the concept of perioperative ERAS, the incidence of surgical complications has decreased significantly. In recent years, the ERAS concept has been mainly used for elective GS in abdominal surgery [10, 11].

Abdominal infection is a common disease in surgical acute abdomen. It is a type of disease in which there are infections in the abdominal cavity, mainly abdominal pain and bloating. Clinically, it is generally divided into local abdominal cavity infection and diffuse abdominal cavity infection. Diffuse abdominal cavity is a severe abdominal cavity infection, most of which have rapid onset, rapid progress, and critical illness, with higher postoperative complications, higher mortality, longer hospital stays, and high hospital costs. It is often accompanied by severe systemic inflammatory response (SIRS) and pathophysiological disorders, often with sepsis or multiple organ dysfunction, and the stress response is relatively severe, requiring early diagnosis and urgent treatment. Patients with severe abdominal infections are admitted to the hospital with a more severe stress metabolic state than general elective GS. If surgical trauma is added at this time, the double blow will aggravate the stress metabolic state of the patient's body. In a short period of time, it may be followed by septic shock and organ failure [12, 13].

The article "Application of Accelerated Rehabilitation Surgery in Gastrointestinal Surgery" was retracted in 2023. Reasons: signs of a paper mill; compromised peer review; unreliable results or conclusions.

#### 2.1.1. Initial Selection of Antibiotics

Start the empirical treatment of antibiotics as soon as possible. Drugs that can cover aerobic bacteria such as intestinal Gram-negative bacilli and Enterococcus and anaerobic bacteria such as fragile Bacteroides should be selected. In order to ensure the effective concentration of drugs, they should be administered intravenously. For severe abdominal infection that endangers the patient's life, the initial treatment of antibiotics must have sufficient intensity.

#### 2.1.2. Adjustment of Drug Use

Relevant samples shall be kept for culture as far as possible before giving antibacterial treatment, and drug sensitivity test shall be carried out after obtaining pathogenic bacteria as the basis for adjustment of drug use.

Accelerating the development of rehabilitation surgery in my country is still in its infancy, mainly due to the current domestic hospitals generally focusing on scale expansion, neglecting benefits, and emphasizing doctor's orders. In this case, exploring a feasible, efficient, feasible, operability, and effective improvement of curative effect and accelerating the construction of rehabilitation surgery centered on adjuvant therapy have become a hot spot in my country's medical community [14, 15].

ARS can shorten the waiting time and cost of patients discharged from the hospital. Speeding up rehabilitation surgery is of great significance to disease diagnosis and evaluation. It can alleviate the pain of patients and improve their confidence and satisfaction in treatment, promote the recovery of the patient's body, and reduce or eliminate adverse emotional reactions. At present, ARS has accumulated rich experience and significant progress. Research reports on ERAS in many major international journals have shown a surge in the past few years. The clinical application of ERAS in various countries has achieved effective results in supporting patient progress, reducing complications, improving patient comfort, accelerating patient recovery, and shortening the length of hospital stay [16, 17].

The article "Application of Accelerated Rehabilitation Surgery in Gastrointestinal Surgery" was retracted in 2023. Reasons: signs of a paper mill; compromised peer review; unreliable results or conclusions.

### 2.2. Perioperative Management of GS

The perioperative period is the key to affecting the quality of life of the patient. In the early stage of the disease, the patient will have serious complications and various physiological and metabolic problems. If it is not controlled, it is easy to cause death. The perioperative period means that the hospital has different treatment methods at different stages when treating patients. Because the patient has great defects in physiology and psychology, it needs to be enlightened before surgery. They need anesthesia to induce and control the patient's entry into the operating room and make it recover smoothly and effectively. At the same time, it can also provide a good rehabilitation environment for patients. Preoperative preparations include the use of observation methods in clinical diagnosis to allow enough time for the patient to complete the examination of the disease and related diseases. And according to the actual situation, choose the appropriate type of operation method with different functions and good curative effect. Preoperative preparations include careful preoperative physical examination, preoperative medication, and treatment of comorbidities. Postoperative treatment includes postoperative complications [18, 19]. Enhance the communication with patients and their families, and explain clearly to patients and their families about the patient's condition, diagnosis, operation method, necessity of operation, effect of operation, possible complications and preventive measures, risk of operation, recovery process, and recovery after operation, so as to obtain trust and cooperation and make patients accept operation happily. Fully respect the patient's independent choice. Diagnostic and treatment measures should be taken on the premise of the patient's “informed consent.” If the patient has no informed consent, it is not suitable to do any operation or damaging treatment.

The ERAS group needs to provide preoperative education and psychological counseling to the patients and their families when they are admitted to the hospital. Fasting for 6 hours before surgery, intravenous general anesthesia is selected as an anesthesia method, and anesthetic drugs that can promote postoperative recovery are used. During the operation, the patient is covered with thermal insulation blankets or clothing to maintain body temperature. If necessary, a hot water bottle or electric heater can be added to monitor the body temperature. In the perioperative period, restrictive fluid replacement is used to control the amount of fluid infusion. A small amount of water can be started 6 hours after waking up from anesthesia and gradual transition to general food; otherwise, the observation period will be extended. Encourage patients to exercise appropriately at the bedside on the first day after surgery. If the patient has upper abdominal pain, indomethacin suppository can be used for analgesia.

The article "Application of Accelerated Rehabilitation Surgery in Gastrointestinal Surgery" was retracted in 2023. Reasons: signs of a paper mill; compromised peer review; unreliable results or conclusions.

The perioperative treatment measures of the traditional treatment group are mainly based on the ERCP diagnosis and treatment guidelines. For the parts that are not clearly stated in the guidelines, the previous clinical routine treatment methods shall prevail. The preoperative fasting time is 12 hours, and the water-free time is 8 hours. The anesthesia method is intravenous general anesthesia, and there are no special requirements for anesthesia medication. During the perioperative period, an open rehydration strategy was used to adequately replenish fluids. There are no strict requirements for the patient's early bed or bedside activities. The treatment of upper abdomen discomfort after the operation is mainly antispasmodic, and analgesia is not routinely performed. Do not contact infected patients. Prevent personnel with upper respiratory tract infection from entering the operating room (prophylactic use of antibiotics): (1) operations involving infectious lesions or incision close to the infected area, (2) gastrointestinal surgery, (3) major surgery with long operation time, (4) contaminated trauma, long debridement time, or difficult to completely debridement, (5) cancer surgery, (6) cardiovascular surgery, (7) artifact implantation, and (8) organ transplantation.

### 2.3. Gastrointestinal Surgery

The stomach and intestines are very delicate parts. If you do not pay attention to maintenance, it is easy to suffer from gastrointestinal diseases. Nowadays, young people are too busy at work and often do not pay attention to their diet, neglecting the ability of their stomachs. I like to eat some spicy and irritating foods. As a result, it is easy to cause gastrointestinal diseases for a long time.

GS mainly treats diseases of the stomach, pancreas, small intestine, large intestine, and other organs. Some hospitals do not perform GS alone but classify it as general surgery. GS is an important part of general surgery. In recent years, GS has made great progress.

#### 2.3.1. The Difference between GS and Gastroenterology

One is surgery, and the other is internal medicine. For example, if you have indigestion, you need to go to the digestive department. If it is a disease of the digestive system, surgery is needed. No matter what the disease is, it should be prevented as soon as possible. Gastrointestinal diseases are mainly caused by improper diet. Do not eat too often even in the hot summer; usually after stomach irritation, some people will get sick in winter. Moreover, staying up late or skipping breakfast can also cause great damage to the stomach, so try to avoid it.

The article "Application of Accelerated Rehabilitation Surgery in Gastrointestinal Surgery" was retracted in 2023. Reasons: signs of a paper mill; compromised peer review; unreliable results or conclusions.

#### 2.3.2. Gastrointestinal Disease

As a common disease among Chinese residents, digestive tract diseases seriously endanger the health and quality of life of residents. In recent years, the incidence of gastrointestinal diseases has increased significantly. With the change of people's eating habits and the increase of social pressure, the population of gastrointestinal diseases is getting younger and younger. At present, the first and most effective treatment method for gastrointestinal diseases is surgical treatment, the purpose of which is to remove the lesions, ensure smooth drainage, and relieve obstruction. However, the biliary system has a complex anatomical structure, special physiological functions, diverse pathological and clinical manifestations, and large surgical trauma. Therefore, the perioperative care of biliary surgery is risky and challenging. The traditional perioperative care measures implemented in the past have caused medical staff to face many problems, such as slow postoperative recovery, many complications, severe postoperative pain and long time, and high hospitalization costs. In view of this, domestic and foreign medical staff have made unremitting efforts to develop a more optimized and perfect perioperative care plan to make up for the shortcomings of traditional nursing measures, reduce the incidence of complications, improve the pain status of patients, and shorten the length of hospitalization. Save hospitalization costs, improve comfort experience, accelerate postoperative recovery, and improve the quality of life.

The combination of traditional Chinese and Western medicine can reduce the adverse reactions of Western medicine and improve the good compliance of patients. In the treatment of difficult gastrointestinal diseases, the mutual mechanism of integrated traditional Chinese and Western medicine is used to achieve the purpose of high cure rate. The prospect of integrated traditional Chinese and Western medicine in the treatment of gastrointestinal diseases should develop to a scientific system with high standards, strict requirements, openness, diversification, and sustainable development and strengthen “pertinence”, “individualization,” and “comprehensiveness.” Only when integrated traditional Chinese and Western medicine in the treatment of gastrointestinal diseases can we make a breakthrough and give full play to the advantages of syndrome differentiation and treatment of Western medicine and traditional Chinese medicine. Traditional Chinese medicine is broad and profound. Using the combination of Chinese and Western medicine to treat gastrointestinal diseases can take the advantages of Chinese and Western medicine and avoid their disadvantages, which is of positive significance to the treatment of gastrointestinal diseases.

The article "Application of Accelerated Rehabilitation Surgery in Gastrointestinal Surgery" was retracted in 2023. Reasons: signs of a paper mill; compromised peer review; unreliable results or conclusions.

### 2.4. Economic Benefits in Accelerated Rehabilitation Surgery

ERAS optimizes perioperative treatment measures to achieve low risk and reduce pain as surgical goals. ERAS treatment covers the entire surgical process including preoperative patient education, surgical decompression, pain management, and ERAS team building. In the specific implementation process, focus on promoting the effective recovery of patients in terms of incision selection, instrument use, and incision suture.

#### 2.4.1. Cost

Cost refers to all human and material resources used to perform a specific treatment or intervention. Direct costs refer to medical and non-medical costs directly related to the treatment of a patient's disease. Indirect costs are loss caused by illness, reduced or absent from work or even death, and the cost of patients' family members absent from work due to “support.” Work is calculated based on social value. The calculation formula is as follows:

(1) $$\begin{array}{c} \text{Indirect cost}=\left(\text{NDMWP}+\text{NDAFM}\right)\times \text{ASDW}. \end{array}$$

Among them, NDMWP is the number of days lost by the patient, NDAFM is the number of days lost by the accompanying family member, and ASDW is the average daily wage in society.

#### 2.4.2. Cost Evaluation

Incremental analysis is an important analysis method in cost-benefit analysis. When changing from one treatment plan to another, the cost and result of the change will be calculated, and then, the ICER rate will be calculated. Each ICER value runs between two different processing options. The formula is as follows:

(2) $$\begin{array}{c} \text{ICEP}=\frac{A_{1}-A_{2}}{B_{1}-B_{2}}=\frac{\Delta A}{\Delta B}. \end{array}$$

## 3. Experimental Method

### 3.1. Experimental Objectives

ARS is used in clinical departments such as GS to comprehensively analyze the postoperative effect indicators and patient cost indicators and study the effect and value of accelerated rehabilitation operations. Select three surgical indicators of radical gastric cancer, radical resection of colorectal cancer, and treatment of abdominal infection to quantify the efficacy and cost-effectiveness, and provide a factual basis for use and promotion.

### 3.2. Target Disease Selection

#### 3.2.1. Gastric Cancer

Gastric cancer is a malignant tumor that originates from the epithelium of the stomach lining. Intestinal obstruction, abdominal hemorrhage, duodenal stump fistula, and anastomotic fistula after radical gastric cancer surgery are the main complications. Surgery for gastric cancer is traumatic, and the scope of tissue resection is wide. In addition, traditional perioperative interventions such as bowel preparation, excessive fluid infusion, and use of opioid analgesics will prolong the patient's postoperative recovery to a certain extent. The early recovery of gastrointestinal function after radical gastric cancer can help reduce the incidence of postoperative complications and postoperative hospital stay. The application of ARS in the treatment of gastric cancer includes the following: preoperative education, bowel preparation, and carbohydrate use; reasonable intraoperative anesthesia, restricted fluid infusion, and fine and minimally invasive surgery; and effective postoperative pain relief methods and early activities and eating. The incidence rate of gastric cancer is obviously different from that in the south. The incidence rate of distal gastric cancer is high in the long-term consumption of smoked and salted foods and is related to the high content of carcinogens or carcinogens in food such as nitrite, mycotoxins, and polycyclic aromatic hydrocarbons. The risk of gastric cancer in smokers is 50% higher than that in nonsmokers.

The article "Application of Accelerated Rehabilitation Surgery in Gastrointestinal Surgery" was retracted in 2023. Reasons: signs of a paper mill; compromised peer review; unreliable results or conclusions.

#### 3.2.2. Colorectal Cancer

Colorectal cancer is a colorectal epithelial tumor that penetrates the muscularis mucosa and infiltrates the submucosa. It is a common malignant tumor of the digestive tract and the second largest tumor of the digestive tract. Colon cancer is a common malignant tumor in my country. It ranks fourth among malignant tumors in my country, and it is on the rise.

#### 3.2.3. Abdominal Infection

Abdominal infection is a common disease in surgical acute abdomen. It is a type of disease in which there are infections in the abdominal cavity, mainly abdominal pain and bloating. Clinically, it is generally divided into local abdominal cavity infection and diffuse abdominal cavity infection. Diffuse abdominal cavity is a severe abdominal cavity infection, most of which have rapid onset, rapid progress, and critical illness, with higher postoperative complications, higher mortality, longer hospital stays, and high hospital costs. It is often accompanied by severe systemic inflammatory response (SIRS) and pathophysiological disorders, often with sepsis or multiple organ dysfunction, and the stress response is relatively severe, requiring early diagnosis and urgent treatment. Patients with severe abdominal cavity infection are in a more severe metabolic state than general elective GS when they are admitted to the hospital.

The article "Application of Accelerated Rehabilitation Surgery in Gastrointestinal Surgery" was retracted in 2023. Reasons: signs of a paper mill; compromised peer review; unreliable results or conclusions.

### 3.3. Inclusion Criteria and Exclusion Criteria

#### 3.3.1. Inclusion Criteria

The inclusion criteria are as follows:

1. Patients are diagnosed with severe abdominal cavity infection and undergo emergency surgery and are older than 14 years old
2. Patients are diagnosed with colorectal cancer (PG-SGA score ≥ 4 points); the operation method is laparoscopic-assisted radical resection of colorectal cancer
3. The preoperative gastroscopy biopsy confirmed the pathological diagnosis, and the preoperative auxiliary examination did not indicate distant metastasis and the third station lymph node metastasis
4. No distant metastases such as brain, lung, liver, and spleen were found before operation
5. Preoperative assessment of cardiopulmonary function can tolerate surgery
6. There are no acute intestinal obstruction, perforation, and hemorrhage
7. There is no radiotherapy, chemotherapy, or traditional Chinese medicine treatment before operation
8. Patients are informed of this study and sign an informed consent form

#### 3.3.2. Exclusion Criteria

The exclusion criteria are as follows:

1. People with severe cognitive impairment
2. The patient who died within 24 hours of admission
3. History of severe cardiovascular and cerebrovascular diseases, severe liver and kidney and other organ dysfunction, pregnancy, or mental illness
4. Preoperative gastrointestinal obstruction, tumor perforation, and severe bleeding excluded
5. Having a history of abdominal surgery, hypertension, or diabetes
6. The patient or family members disagreeing with this trial study

### 3.4. Experiment Grouping

Patients were screened according to the inclusion criteria. The patients selected in this article are all patients from the People's Hospital of the city. A total of 150 patients with gastric cancer, colorectal cancer, and abdominal infection were screened out. These patients will be admitted from January 1 to July 31, 2021. The patients will be numbered, the single number will be treated with traditional methods, and the even number will be treated with ARS. There are 75 people in each group. Patients and their families signed an informed consent form before the operation.

### 3.5. Observation Indicators

The preoperative data of the two groups of patients were recorded: age, gender, body weight, BMI, and serum albumin level one day before the operation. The following are the surgery-related indicators: operation time, intraoperative blood loss, postoperative bowel function recovery time, hospital stay, and perioperative complications. The following are the biochemical indicators: changes in serum PCT, CRP, and PA levels before and after surgery.

The article "Application of Accelerated Rehabilitation Surgery in Gastrointestinal Surgery" was retracted in 2023. Reasons: signs of a paper mill; compromised peer review; unreliable results or conclusions.

### 3.6. Perioperative Management

#### 3.6.1. Speed Up the Treatment of the Rehabilitation Group

*(1) Preoperative Publicity and Education*. Advise patients to actively exercise cardiopulmonary function before surgery, encourage patients to eat as soon as possible after surgery, and advise patients to exercise as soon as possible with the help of the patient's family or other people. Observe preoperative bowel preparation. In the working group applying the concept of ARS, there is no systematic mechanical dissection of the intestines, and only enema is performed before surgery and the morning before surgery when necessary.

*(2) Reasonable Choice of Anesthesia Plan*. You can choose a more sensible anesthesia method and an anesthesia method that is beneficial to the patient according to the specific situation of the patient, which can not only reduce the burden on the heart and kidneys but also protect the patient's respiratory function to a certain extent. Try to keep the patient's body temperature stable during the operation. Hypothermia is a common complication of surgery. During the operation, monitor the patient's body temperature, pay attention to maintaining body temperature, inject warm liquid, raise the temperature of the operating room, and rinse with warm water. Pay attention to the amount of fluid during surgery, and use drugs to control the contraction and expansion of blood vessels to help maintain the stability of blood pressure

*(3) Postoperative Pain Relief*. In terms of postoperative analgesia, patients in the accelerated rehabilitation group used self-guided analgesic pumps for analgesia, combined with other analgesics that have less impact on digestive function as auxiliary analgesia. Eat and exercise as soon as possible after the operation. If the patient's condition permits, an appropriate amount of 10% glucose 200 ml can be taken 8 hours after the operation, and the dosage should be gradually increased according to the specific situation. The patient is encouraged to get up and carry out activities after the operation to help the patient develop an appropriate activity plan. Encourage patients to achieve the goal of getting up every day. Check the amount of liquid injected. Appropriate fluid replacement therapy will be performed before and after the operation. In ARS, excessive fluid supplementation during the perioperative period is not recommended. The operator shall carefully check the patient's name, gender, medical record number, bed number, diagnosis, operation site, and operation room. Patients must remove dentures before entering the operating room, and valuables shall be kept by their families. The members of the operation team participating in the operation on the same day shall enter the operating room in advance, and the operator shall tell the important steps, possible accident countermeasures, and strictly implement the operation plan formulated through preoperative discussion and the requirements of operation safety check. During the operation, anesthesiologists shall always monitor patients and shall not leave their posts without authorization

The article "Application of Accelerated Rehabilitation Surgery in Gastrointestinal Surgery" was retracted in 2023. Reasons: signs of a paper mill; compromised peer review; unreliable results or conclusions.

#### 3.6.2. Control Group Treatment

1. No solid food is allowed 12 hours before the operation, and drinking water and other beverages are not allowed 4 hours before the operation. Before the operation begins, the patient will be placed with a catheter and a gastric tube
2. In intraoperative general anesthesia, the patient's body temperature changes are not monitored in real time. Intraoperative fluid infusion is mainly to maintain blood pressure and increase blood volume. Drainage tubes are routinely placed during surgery
3. In postoperative pain relief, an analgesic pump is not routinely placed to relieve pain, and analgesic drugs are used according to the patient's pain. The main basis for eating is the patient's exhaust. If there is no abnormal urination, remove the catheter after 3 days

## 4. Results

### 4.1. Comparison of General Information of the Two Groups of Patients

According to the collected patients, the brief statistical results of this article are shown in Table 1. This table mainly shows the age, gender, and distribution of the three diseases of the patients in the accelerated group and the control group.

As shown in Figure 1, we can judge that among the patients, the age is generally over fifty-five years, and the number of males is the same as that of females. The most afflicted is gastric cancer, followed by rectal cancer and finally abdominal infection.

### 4.2. Safety Comparison

According to the experimental investigation and some conditions during and after the operation, this article compares and analyzes the operation time, intraoperative blood loss, exhaust time, and the number of days in the hospital after the operation and draws the data in Table 2.

As shown in Figure 2, we can find that in the accelerated group, the average operation time is about 160 minutes, while the time in the control group is relatively shorter. However, the postoperative exhaust time and hospital rest days in the accelerated group were much shorter than those in the control group. This shows that the effect of ARS is better than traditional methods.

### 4.3. Comparison of Postoperative Complications

According to the survey, we obtained the following data after returning to the patients. In the return visit of patients, postoperative complications occurred, including incision infection, lung infection, anastomotic leakage, and intestinal obstruction. The specific data are shown in Table 3.

The article "Application of Accelerated Rehabilitation Surgery in Gastrointestinal Surgery" was retracted in 2023. Reasons: signs of a paper mill; compromised peer review; unreliable results or conclusions.

As shown in Figure 3, we can see that in the accelerated group, the number of postoperative infections is smaller than that in the control group. And the *P* value is less than 0.05, which is statistically significant.

### 4.4. Evaluation of Clinical Efficacy

According to the results of the survey, among patients with gastric cancer, colorectal cancer, and abdominal infections, the groups receiving accelerated rehabilitation surgical treatment and traditional treatment have different curative effects. The specific situation is shown in Table 4.

As shown in Figure 4, we can see that the left picture is the treatment situation of the accelerated group, and the right picture is the average level of curative effect of the traditional treatment group. From the comparison in the figure, we find that the number of people in the accelerated treatment group with obvious treatment effect is more than that in the traditional treatment group, and there are more people who have the effect. The traditional group has more invalids than the accelerated group. This shows the effectiveness of the accelerated treatment.

## 5. Conclusion

Improving the quality of medical services and improving the treatment effect of surgical patients are issues that surgeons have been paying attention to and thinking about. Aiming at the role of ARS in gastrointestinal patients, this article applied the concept of accelerated rehabilitation surgery (ARS) to the perioperative care of gastrointestinal patients. And it was observed that compared with conventional nursing measures, the recovery of gastrointestinal function, waking up early, hospitalization days, total hospitalization expenses, complication rate, and pain were observed. To test the safety, effectiveness, and feasibility of applying the concept of rapid rehabilitation surgery to patients and to provide theoretical basis and clinical practice experience for the application of gastrointestinal patients in the perioperative period, this paper proposes that it can promote better treatment effects, shorter hospital stays, and lower costs. Moreover, according to the return visit records, it can be found that the probability of postoperative infection of patients is smaller in ARS. All experimental results show that ARS has a distinct impact in the treatment of gastrointestinal diseases.

## Figures and Tables

**Figure 1:** Comparison of the general data between the two patient groups.

The article "Application of Accelerated Rehabilitation Surgery in Gastrointestinal Surgery" was retracted in 2023. Reasons: signs of a paper mill; compromised peer review; unreliable results or conclusions.

**Figure 2:** Security comparison of two groups.

**Figure 3:** Comparison of postoperative complications.

**Figure 4:** Clinical efficacy evaluation.

**Table 1:** Comparison of the general data between the two patient groups.

Clinical factors	Accelerated group	Control group	Variance
Age	56.42	56.31	0.12
Female	39	36	0.003
Male	38	37	0.005
Stomach	30	28	0.173
Colorectal	26	25	0.179
Abdominal cavity	21	20	0.185

**Table 2:** Security comparison of two groups.

	Accelerated group	Control group	*t* value	*P* value
Operation time	160	155	0.8	0.4
Intraoperative bleeding	60	58	0.2	0.8
Exhaust time	2.6	4.9	-10	0
Postoperative hospital stay	7.5	12	-16	0

**Table 3:** Comparison of postoperative complications.

	Accelerated group	Control group	*P* value
Incision healed poorly	2	4	0.032
Lung infection	1	2	0.025
Anastomotic fistula	0	1	0.02
Intestinal obstruction	1	3	0.031

**Table 4:** Clinical efficacy evaluation.

	Accelerated group		Control group	
	Example number	Efficacy rate	Example number	Efficacy rate
Show effect	20	26.7%	15	20%
Valid	30	40%	25	33.3%
Invalid	25	33.3%	35	46.7%

## Data Availability

The data underlying results presented in the study are available within the manuscript.

## References

[1] Laizhi Y., Yin F., Yan P. (2020). To explore the clinical effect of no gastrointestinal decompression in the treatment of acute pancreatitis based on the concept of accelerated rehabilitation surgery. *Journal of Clinical Emergency Medicine*.

[2] Weiwei X., Yuli A. (2019). Application progress of accelerated rehabilitation surgery concept in gastrointestinal surgery. *Digest of World Latest Medical Information*.

[3] Qin L. (2019). Observation on the effect of accelerated rehabilitation surgery in patients with gastric cancer in gastrointestinal surgery. *Forum on Primary Medicine*.

[4] Mingxu S., Zhiping C., Haiyan W. (2020). Research on the application value of the concept of accelerated rehabilitation surgery in the nursing management of gastrointestinal surgery. *Chinese Health Industry*.

[5] Jian S., Linhao C., Fangqin X. (2019). Application analysis of the concept of accelerated rehabilitation surgery in common emergency operations in gastrointestinal surgery. *Fujian Medical Journal*.

[6] Changqing J., Jinshen W. (2019). The important role of accelerated rehabilitation surgery in the application of evidence-based medicine in gastrointestinal surgery. *Journal of Shandong University (Medical Edition)*.

[7] Guoqiang D., Nan Z., Haicheng Y. (2021). Application of accelerated rehabilitation surgical path in the perioperative period of laparoscopic incisional hernia repair. *Chinese Journal of General Surgery*.

The article "Application of Accelerated Rehabilitation Surgery in Gastrointestinal Surgery" was retracted in 2023. Reasons: signs of a paper mill; compromised peer review; unreliable results or conclusions.

[8] Xiaoqing Z., Qingxian K., Jin G. (2020). Application research of accelerated rehabilitation surgical nursing in elderly laparoscopic radical gastrectomy. *Contemporary Nurses (Academic Edition)*.

[9] Kangwen C., Guihe W., Aiping T. (2020). Application of the concept of accelerated rehabilitation surgery in laparoscopic-assisted radical gastric cancer surgery in elderly patients. *Chinese Journal of Multiple Organ Diseases in the Elderly*.

[10] Shangjie X., Wenyi Y., Lu X. (2019). Application of minimally invasive surgery and early postoperative feeding in the accelerated rehabilitation of neonatal duodenal obstruction. *Journal of Clinical Pediatric Surgery*.

[11] Peng J., Qi G., Xuefei Q. (2019). Application of multimodal analgesia in patients undergoing gastrointestinal tumor surgery in accelerated rehabilitation surgery. *Shanghai Medical Science*.

[12] Chen J., Luo B., Huang J., Wang R., Hu M. (2020). Application of the concept of accelerated rehabilitation surgery in the teaching of gastrointestinal surgery. *Chinese Continuing Medical Education*.

[13] Li X. (2020). Application value of accelerated rehabilitation surgery in patients with gastrointestinal tumor surgery. *Journal of Qiqihar Medical College*.

[14] Haotang W., Wang Jialei W., Gang X. (2019). Clinical study on the early recovery effect of NOSES in patients with colorectal cancer in accelerated rehabilitation surgery. *Colorectal and Anal Surgery*.

[15] Wensheng L., Wenyan X., Shunrong J. (2019). Application experience of accelerated rehabilitation surgery concept in the perioperative period of laparoscopic pancreatic body and tail resection. *Journal of Laparoscopic Surgery*.

[16] Shudi Y., Yuli Z., Ling L. (2020). Application and prospect of accelerated rehabilitation surgery in neonatal perioperative management. *Journal of Kunming Medical University*.

[17] Xiaoping G., Ju W., Hongwei J. (2020). Application of accelerated rehabilitation surgery in laparoscopic repair of giant gastroduodenal ulcer perforation. *Chinese Journal of General Surgery (Electronic Edition)*.

[18] Wenting H., Fangchan X., Zhen L. (2019). Application of minimally invasive surgery and early postoperative feeding in the accelerated rehabilitation of neonatal duodenal obstruction. *Journal of Clinical Pediatric Surgery*.

[19] Huang W., Xu F., Liu Z. (2019). The effect of accelerated rehabilitation surgery on the nursing effect and sleep time of patients with rectal cancer and diabetes. *World Journal of Sleep Medicine*.

